# Identification of Hub Genes of Keloid Fibroblasts by Coexpression Network Analysis and Degree Algorithm

**DOI:** 10.1155/2022/1272338

**Published:** 2022-01-10

**Authors:** Xianglan Li, Rihua Jiang, Haiguo Jin, Zhehao Huang

**Affiliations:** ^1^Department of Dermatology, China-Japan Union Hospital of Jilin University, Changchun 130033, Jilin, China; ^2^Department of Radiotherapy, Jilin Guowen Hospital, Changchun 130000, Jilin, China; ^3^Department of Neurosurgery, China-Japan Union Hospital of Jilin University, Changchun 130033, Jilin, China

## Abstract

**Background:**

Keloid is a benign dermal tumor characterized by abnormal proliferation and invasion of fibroblasts. The establishment of biomarkers is essential for the diagnosis and treatment of keloids.

**Methods:**

We systematically identified coexpression modules using the weighted gene coexpression network analysis method (WGCNA). Differential expressed genes (DEGs) in GSE145725 and genes in significant modules were integrated to identify overlapping key genes. Gene Ontology (GO) and Kyoto Encyclopedia of Genes and Genomes (KEGG) enrichment analyses were then performed, as well as protein-protein interaction (PPI) network construction for hub gene screening.

**Results:**

Using the *R* package of WGCNA, 22 coexpression modules consisting of different genes were identified from the top 5,000 genes with maximum mean absolute deviation in 19 human fibroblast samples. Blue-green and yellow modules were identified as the most important modules, where genes overlapping with DEGs were identified as key genes. We identified the most critical functions and pathways as extracellular structure organization, vascular smooth muscle contraction, and the cGMP-PKG signaling pathway. Hub genes from key genes as BMP4, MSX1, HAND2, TBX2, SIX1, IRX1, EDN1, DLX5, MEF2C, and DLX2 were identified.

**Conclusion:**

The blue-green and yellow modules may play an important role in the pathogenesis of keloid. 10 hub genes were identified as potential biomarkers and therapeutic targets for keloid.

## 1. Introduction

Keloids are mainly associated with excessive proliferation of fibroblasts and massive deposition of the extracellular matrix following skin injury [1]. The clinical presentation of keloids is primarily a growth of scar tissue above the skin, usually accompanied by pruritus and pain [2]. Some studies have shown that keloid formation is closely related to genetic regulation, inflammatory factors, cytokines, and immune factors [3, 4]. The treatment of keloid is not ideal because of unclear pathogenesis and regulatory mechanisms underlying keloids [5]. For these reasons, the identification of hub genes involved in keloid is urgent and highly demanded for improving the clinical outcome.

Keloids have some similarities to tumors; in particular, the fibroblasts in keloids have unlimited proliferation and invasive growth [6]. Fibroblasts are the most abundant cells in the dermis and maintain dermal structure by producing an extracellular matrix (ECM) [7]. The ECM is in a constant state of synthesis, degradation, and remodeling, both under normal conditions and in the presence of disease or injury [8]. After a 2-3 d period of haemostasis and inflammation, the dermis undergoes a proliferative phase in which fibroblasts move from a homeostatic state to an activated state, where their ability to proliferate and migrate is significantly enhanced and they differentiate into a unique phenotype, myofibroblasts, which have stronger contractile properties and synthesized the ECM more rapidly, thereby accelerating wound closure [9]. Once the tissue is fully repaired, these myofibroblasts undergo apoptosis and senescence or revert to deactivated fibroblasts [10]. However, the persistence of active fibroblasts (including myofibroblasts) at the site of injury may lead to excessive deposition of the ECM and the formation of abnormal scarring. So, the thickness of the scar is usually positively correlated with the number of fibroblasts in the dermis and the density of collagen (the main component of the ECM). Therefore, inhibition of fibroblast proliferation has long been a hot topic in scar research.

Weighted gene coexpression network (WGCNA) analysis [11] first clusters genes with similar expression patterns into a module by calculating expression correlations between genes and then analyses the correlation between the module and the sample characteristics, such as clinicopathological parameters and treatments. WGCNA rapidly extracts modules and genes that correlate with sample characteristics from transcriptomic data and obtains biomarkers with better biological significance than differential expression analysis based on comparative intramodule connectivity and gene significance [12]. In this study, we constructed a WGCNA-based gene coexpression network, identifying 22 modules. We also performed GO and KEGG enrichment analysis of genes overlapping in 2 modules closely related to keloid fibroblast and DEGs. A PPI network was also constructed, and 10 hub genes were screened out, including BMP4, MSX1, HAND2, TBX2, SIX1, IRX1, EDN1, DLX5, MEF2C, and DLX2. These hub genes may be biomarkers for diagnosis and therapy of keloid.

## 2. Methods

### 2.1. Data Collection

The gene expression dataset GSE145725 (https://www.ncbi.nlm.nih.gov/geo/query/acc.cgi?acc=GSE145725) provided by Yuanyuan Kang et al. [13] was downloaded from the Gene Expression Omnibus (GEO) database [14]. 10 cell lines (5 normal fibroblast and 5 keloid fibroblast) were grown in replicate cultures and subjected to RNA extraction. One of the keloid samples was removed after QC. RNA samples with RNA integrity number (RIN) above 9.8 were hybridized to GeneChip PrimeView Human Gene Expression Arrays (Affymetrix).

### 2.2. Weighted Gene Correlation Network Analysis (WGCNA)

WGCNA aims to identify coexpressed gene modules to explore the relationship between gene networks and phenotypes and to examine the core genes in the network [11]. Only top 5000 genes with maximum mean absolute deviation were selected, and abnormal samples were detected using the Z-score method, with Z-score value −2.5 as a cutoff for identifying outliers. According to the scale-free topology criterion, 22 was determined as the optimal soft threshold, with minimum module size 30 and the module detection sensitivity deep split 2. Based on the soft threshold, scale-free network and topology matrices were constructed. The gene modules were dynamically cut and eigengenes were calculated, with 30 as the minimum number of genes in the module. According to the module eigengenes, intermodule correlations were constructed and hierarchical clustering was performed. Finally, 22 modules were obtained and Pearson correlations between modules and clinical features were analyzed.

### 2.3. Differential Expression Analysis

The GSE145725 dataset was downloaded from the GEO database via the *R* (version 3.6.3) package of GEO query 2.54.1 [15]. The probes corresponding to more than one molecule were removed, and only the probe with the largest signal value was retained when probes correspond to the same molecule. Then, the samples were normalized by box plots, and the clustering between sample groups was demonstrated by PCA plots and UMAP plots. The limma 3.42.2 package was then used for the differential expression analysis between the keloid fibroblast group and normal fibroblast. The top 20 differentially expressed genes (DEGs) were visualized as heatmap using the ComplexHeatmap 2.2.0 package [16] with the clustering method of Euclidean distances.

### 2.4. Key Gene Identification and Enrichment Analysis

The green-yellow and blue modules are the modules most associated with the keloid fibroblast phenotype. The overlapped genes in the two modules and DEGs were identified as the key genes. Using the org.Hs.eg.db 3.10.0 package, the key gene symbols were converted into Entrez IDs and then subjected to Gene Ontology (GO) and Kyoto Encyclopedia of Genes and Genomes (KEGG) enrichment analysis through the cluster Profiler 3.14.3 package [17].

### 2.5. Protein-Protein Interaction (PPI) Network Construction

Key genes were uploaded to the STRING database (version 11.0) to construct the PPI network [18]. Interactions with a score above 0.4 were considered significant. The PPI network was visualized using Cytoscape software (version 3.8.3) [19]. Top 10 key genes with highest degree were detected as hub genes by CytoHubba plugin.

### 2.6. Correlation Analysis and Expression of Hub Genes

Correlations between hub genes were analyzed, and Spearman's correlation coefficients were calculated for variables that did not satisfy the normal distribution (*P* < 0.05). The correlation matrix and scatter plot were also plotted using the ggplot2 3.3.3 package.

The expression profiles of the hub genes were first subjected to the Shapiro–Wilk normality test. The Wilcoxon rank sum test was chosen when the gene expression values did not satisfy the normality test (*P* < 0.05).

## 3. Results

### 3.1. WGCNA

To identify significant modules, firstly, expression profile distribution of all samples was checked and abnormal samples were detected. The results showed that the median across the samples was essentially at one level, indicating good normalization between samples (Figure 1(a)). Besides, no outlier sample was found (Figure 1(b)). Then, all given soft powers were traversed to get the smallest one which can make the correlation network conform to nonscale network attributes, and a soft threshold of 22 was chosen (Figure 1(c)). Based on the soft threshold power and dynamic tree cut, 22 modules were identified (Figure 2(a)). To clarify the interrelationship between the 22 coexpression modules, we performed a cluster analysis (Figure 2(b)). 22 modules differed significantly from each other (Figure 2(c)). Several modules were associated with keloid fibroblasts. In particular, the blue module was most positively correlated with keloid fibroblasts, and the green-yellow module was the most negatively correlated with keloid fibroblasts.

### 3.2. Differential Expression Analysis

Meanwhile, we performed differential expression analysis on the GSE145725 dataset to identify aberrantly expressed genes in keloid fibroblasts. Principal component analysis (PCA) plots showed significant differences between the keloid fibroblast and normal fibroblast groups (Figure 3(a)). Subsequently, 19043 genes were filtered. Of these, 458 IDs met the threshold of |log2(FC)| > 1 and p.adj<0.05, under which the number of upregulated gene in keloid fibroblasts was 215 and in normal fibroblasts was 243 (Figure 3(b)). In addition, we show the expression profile of top 20 genes with high and low expression in a heat map (Figure 3(c)).

### 3.3. Key Gene Screening and Enrichment Analysis

From WGCNA modules, we selected the blue module and green-yellow module as the important modules (Figure 4(a)). The genes in these modules were then intersected with DEGs, and the 186 overlapped genes were regarded as key genes (Figure 4(b)). To understanding the functions and pathways in which these genes are involved, GO and KEGG enrichment analysis were performed. Through ID conversion, 176 Entrez ID was filtered. Under the criterion of p.adj<0.05 and *q* value<0.2, there were 537 entries for biological process (BP), 3 entries for molecular function (MF), and 4 entries for KEGG. In GO-BP analysis, a bubble plot showed that key genes were significantly enriched in the regulation of supramolecular fiber organization, extracellular structure organization, extracellular matrix organization, regulation of cell growth, positive regulation of cell cycle, connective tissue development, and extracellular structure organization (Figure 4(c)). Oxidoreductase activity, acting on the CH-NH2 group of donors, oxygen as the acceptor, DNA-binding transcription activator activity, RNA polymerase II-specific, DNA-binding transcription repressor activity, and RNA polymerase II-specific were the significant MF entries (Figure 4(d)). Besides, key genes were involved in the vascular smooth muscle contraction, cGMP-PKG signaling pathway, renin secretion, and AGE-RAGE signaling pathway in diabetic complications (Figure 4(e)). There were no GO-CC enrichment terms.

### 3.4. Hub Gene Identification

To find the hub genes in keloid fibroblasts, we uploaded the 186 key genes to the String database. Under the threshold of 0.4 interaction score, a PPI network was constructed (Figure 5(a)). Then, the interaction data were downloaded and imported into Cytoscape software. Filtered by CytoHubba calculation, the top 10 hub genes with highest degree were BMP4, MSX1, HAND2, TBX2, SIX1, IRX1, EDN1, DLX5, MEF2C, and DLX2 (Figure 5(b)). Then, we calculated the correlation of hub gene expression with Spearman's rank (rs) test. There was a positive correlation between BMP4 and MSX1, between MSX1 and SIX1, between HAND2 and EDN1, between HAND2 and DLX5, between HAND2 and DLX2, and between DLX5 and DLX2. Additionally, IRX1 was negatively correlated with HAND2. MEF2C was negatively correlated with SIX1, EDN1, and DLX5 (Figures 6(a) and 6(b)). In terms of expression level, BMP4, MSX1, TBX2, SIX1, DLX5, and DLX2 were lowly expressed, while HAND2, IRX1, EDN1, and MEF2C were highly expressed in keloid fibroblasts (Figure 7).

## 4. Discussion

Despite different treatments such as compression therapy, corticosteroid injection, and surgical methods, the recurrence rate of keloids remains high [20]. To identify better treatment targets of keloid, this study used WGCNA analysis, differential expression analysis, and degree algorithm and screened out 10 hub genes associated with keloid fibroblast from the GSE145725 dataset, including BMP4, MSX1, HAND2, TBX2, SIX1, IRX1, EDN1, DLX5, MEF2C, and DLX2.

Among these hub genes, only BMP4 was reported in keloid. As we know, this gene encodes a secreted ligand of the transforming growth factor (TGF)-*β* superfamily of proteins. Ligands of this family bind various TGF-*β* receptors leading to recruitment and activation of SMAD family transcription factors that regulate gene expression [21]. According to the work of Xing Dai et al., activation of the BMP4/Smad signaling pathway may promote transdifferentiation of primary keloid myofibroblasts to adipocyte-like cells [22].

The emergence of myofibroblasts is an inevitable process of tissue repair, and this transdifferentiation process is dependent on signaling through the TGF-*β*1/Smads pathway, whose activation leads to the binding of Smad3 to Smad4 and the initiation of fibrotic genes expression such as ACTA2 [23, 24]. The TGF-*β*1/Smads signaling pathway runs through the entire process of wound healing from the inflammatory phase to the remodeling phase and is one of the major pathways regulating scar formation [25]. BMP4 could facilitate this pathway, thus suggesting the reliability of the results of this study.

In GO-BP-enriched terms shown in the bubble plot, BMP4 was enriched in terms including smooth muscle cell differentiation, regulation of smooth muscle cell proliferation, smooth muscle cell proliferation, and connective tissue development. These BPs were all related to keloid fibroblasts or keloid [26]. In addition to BMP4, other hub genes were also involved in many GO-BP. EDN1, in particular has a regulatory effect on many keloid-related BPs, including regulation of supramolecular fiber organization, myofibril assembly, regulation of smooth muscle contraction, smooth muscle cell differentiation, smooth muscle contraction, regulation of smooth muscle cell proliferation, smooth muscle cell proliferation, regulation of smooth muscle cell migration, smooth muscle cell migration, smooth muscle cell apoptotic process, regulation of smooth muscle cell apoptotic process, regulation of cell growth, positive regulation of cell cycle process, positive regulation of cell cycle, connective tissue development.

Besides, KEGG enrichment analysis showed that the cGMP-PKG signaling pathway was significantly enriched. As we know, this pathway mediates platelet activation, cardioprotection, smooth muscle relaxation, decrease in intracellular free calcium, and reduced cardiac hypertrophy [27]. Importantly, PKG is a protein kinase that when activated by the second messenger cGMP, phosphorylates VASP, thereby promoting cell growth and differentiation [28], and phosphorylates Bad [29] and CREB [30], thereby decreasing the activity of caspase-3 and inhibiting apoptosis.

Although the sample size of this study is not rich enough and there is no external dataset to validate the screening results, this study is still the first to identify key aberrant genes in keloid fibroblast based on the WGCNA algorithm, which provides therapeutic targets for keloid and reference for future research. The limit is that there are not enough solid foundation to support the opinion. Further experiments are still needed to confirm the study.

## 5. Conclusions

The blue-green and yellow modules may play an important role in the pathogenesis of keloid. 10 hub genes were identified as potential biomarkers and therapeutic targets for keloid.

## Figures and Tables

**Figure 1:** Expression data preprocess and soft power detection. (a) Boxplot plus violin plot showing the expression profile distribution of all keloid fibroblasts samples. (b) Hierarchical clustering showing sample correlations and outlier samples. Samples labeled with red bars in the outlier C row are detected potential outlier samples. (c) Network topology for different soft powers. The soft threshold power in the WGCNA was determined based on a scale-free *R*^2^ (*R*^2^ = 0.85).

**Figure 2:** Construction of coexpression modules. (a), WGCNA module plot. Dynamic Tree Cut represents initial modules. Module colors represent final modules. Each branch in the hierarchical tree or each vertical line in color bars represents one gene. Genes not attributed to any module would be colored by grey. (b) Correlation of all identified modules. Each color represents one module. (c) WGCNA module trait correlation plot. Each row represents one module. Each column represents one trait attribute. Blue color represents negative correlation, and red color represents positive correlation.

**Figure 3:** Differential genes' screening on the GSE145725 dataset. (a) PCA plot. (b) Volcano plot, with threshold as |logFC| > 1 & p.adj <0.05. (c) Heatmap visualizing the expression profile of top 20 genes with the highest or lowest expression.

**Figure 4:** Key genes' screening and function prediction. (a) The scatterplot reveals a strong correlation between module membership (MM) and gene significance (GS) in the blue and green-yellow modules. The dot indicates all genes within the modules. (b) The Venn diagram showing key genes. (c) GO-BP enrichment analysis of key genes. (d) GO-MF enrichment analysis of key genes. (e) KEGG enrichment analysis of key genes.

**Figure 5:** PPI network construction. (a) PPI network was constructed based on 186 key genes in the String website, with interaction score 0.4. (b) Top 10 hub genes were identified by degree algorithm in Cytoscape software.

**Figure 6:** Hub gene correlation. Correlation among hub genes was calculated by Spearman's method and visualized as a matrix heat map (a) and scatter plot (b).

**Figure 7:** Hub gene expression. The difference of hub gene expression between the normal fibroblast group and keloid fibroblast group was calculated by the Wilcoxon rank sum test. ^∗∗∗^*P* < 0.001.

## Data Availability

The data used to support this study are available from the corresponding author upon request.
